The article "Human sperm uses asymmetric and anisotropic flagellar controls to regulate swimming symmetry and cell steering" was retracted in 2021. Reasons: unreliable data; unreliable results or conclusions.

# Human sperm uses asymmetric and anisotropic flagellar controls to regulate swimming symmetry and cell steering

**DOI:** 10.1126/sciadv.aba5168

**Published:** 2020-07-31

**Authors:** Hermes Gadêlha, Paul Hernández-Herrera, Fernando Montoya, Alberto Darszon, Gabriel Corkidi

**Affiliations:** 1 Department of Engineering Mathematics, University of Bristol, BS8 1UB Bristol, UK.; 2 Laboratorio de Imágenes y Visión por Computadora, Departamento de Ingeniería Celular y Biocatálisis, Universidad Nacional Autónoma de México, Cuernavaca, Mexico.; 3 Departamento de Genética del Desarrollo y Fisiología Molecular, Instituto de Biotecnología, Universidad Nacional Autónoma de México, Cuernavaca, Mexico.

## Abstract

Flagellar beating drives sperm through the female reproductive tract and is vital for reproduction. Flagellar waves are generated by thousands of asymmetric molecular components; yet, paradoxically, forward swimming arises via symmetric side-to-side flagellar movement. This led to the preponderance of symmetric flagellar control hypotheses. However, molecular asymmetries must still dictate the flagellum and be manifested in the beat. Here, we reconcile molecular and microscopic observations, reconnecting structure to function, by showing that human sperm uses asymmetric and anisotropic controls to swim. High-speed three-dimensional (3D) microscopy revealed two coactive transversal controls: An asymmetric traveling wave creates a one-sided stroke, and a pulsating standing wave rotates the sperm to move equally on all sides. Symmetry is thus achieved through asymmetry, creating the optical illusion of bilateral symmetry in 2D microscopy. This shows that the sperm flagellum is asymmetrically controlled and anisotropically regularized by fast-signal transduction. This enables the sperm to swim forward.

## Teaser

Human sperm create the optical illusion of symmetric swimming in 2D using asymmetric beating in 3D.

## INTRODUCTION

The coordinated motion of eukaryotic cilia and flagella is the archetype of spontaneous wave generation bridging molecular and microscopic scales in nature (*1*). The flagellum is a moving whip-like cellular appendage found on a large variety of eukaryotic organisms and vital for the reproduction of almost all species (*1*, *2*). Up until now, human sperm have been postulated to swim forward by simply moving their flagellum symmetrically from side-to-side (*2*–*8*). Notably, this perception of symmetry has not changed since Leeuwenhoek’s first observations in the 17th century (Fig. 1). This also led to symmetric idealizations of the waveform in three dimensions (3D), often perceived as a conical helix, similar to a widening corkscrew. This appeared to explain, for example, the observed head spinning and helical trajectories with conserved chirality in free-swimming spermatozoa (*4*, *9*–*14*), whereas our understanding of the human sperm beating has been critically limited to 2D microscopy. 2D observations of waveform symmetry have equally led researchers to infer symmetric control hypotheses for the spontaneous wave generation in flagella (*2*, *3*, *15*–*24*), from the tug of war to curvature control, sliding, and the geometric-clutch hypotheses (*15*–*18*, *21*, *22*, *24*).

The article "Human sperm uses asymmetric and anisotropic flagellar controls to regulate swimming symmetry and cell steering" was retracted in 2021. Reasons: unreliable data; unreliable results or conclusions.

**Fig. 1:** The postulation of symmetry has not changed since Leeuwenhoek’s first observations in the 17th century. (**Top**) The flagellar beat is asymmetric in 3D, characterized by a one-sided stroke in each beating plane that rotates with the flagellum. The out-of-plane motion causes the sperm flagellum to roll around the swimming axis (dark blue axis), causing the sperm to move equally on all sides in 3D. This creates the effect of a precessing spinning top, in which head spinning, ω_spin_, around the longitudinal axis of the sperm (yellow axis) occurs at the same time as, and independently of, the flagellar rolling, ω_roll_, around the swimming axis (Supporting Video S2). (**Bottom**) Planar projection of the 3D beat averages out the one-sided asymmetric stroke and creates the optical illusion of bilateral symmetry in 2D microscopy. Symmetry is thus achieved through asymmetry.

The postulation of symmetric beating is, however, in contrast with the abundance of observations showing structural asymmetries within the flagellar scaffold (*2*, *10*, *20*, *23*, *25*–*36*). Asymmetric waves have been reported in murine spermatozoa (*37*, *38*), while a one-sided stroke is commonly observed in *Chlamydomonas* (*23*, *27*–*29*). Ultrastructural anisotropies and asymmetries are intrinsic to mammalian sperm (*2*, *20*, *30*), present at every level, from asymmetric dynein activity (*25*, *26*, *31*, *32*) to atypical centriole (*33*) and an ever growing number of regulatory complexes (*10*, *27*, *29*, *34*–*36*), including anisotropic localization of membrane ion channels, which are critical for sperm capacitation (*10*, *34*). These intrinsic molecular asymmetries must somehow still dictate the flagellar coordination and be manifested in the flagellar beat itself. However, if this is the case, then how does the human sperm flagellum achieve symmetric side-to-side movement and straight-line swimming with asymmetric flagellar controls?

Here, we reconcile molecular and microscopic observations by showing that de facto human sperm use both asymmetric and anisotropic controls to regulate the beat. Spermatozoa roll as they swim (Fig. 1 and movie S2); thus, we used high-speed 3D microscopy to describe the sperm beating, as observed from a frame of reference that moves and rotates with the sperm in 3D, as illustrated by each plane rotation in Fig. 1. Two coactive transversal controls regulate the flagellar beat: (i) An asymmetric traveling wave creates a one-sided stroke, and (ii) an out-of-plane pulsating wave gradually rolls the sperm flagellum so that it beats equally on all sides in 3D. Symmetry is achieved through asymmetry, enabling sperm to swim forward. This creates the effect of a “precessing spinning top,” in which the head spins, “drilling into the fluid,” at the same time as, and independently of, the sperm flagellum rolling around the swimming axis (Fig. 1 and movie S2). The flagellar rolling motion averages out the beat asymmetry and creates the optical illusion that the flagellum moves symmetrically from side to side when observed with 2D microscopy, rendering this intrinsic beat asymmetry invisible until now (Fig. 1). This affects the modulation of curvature, the waveform torsion, and the chirality of the beat via “flagellar perversions.” We suggest that molecular motors are asymmetrically controlled and are, themselves, anisotropically regulated by fast signal transduction along the sperm flagellum. The latter resolves the long-standing paradox by explaining how human sperm can both operate asymmetrically and achieve forward swimming through what appears to be a symmetric movement in 2D.

The article "Human sperm uses asymmetric and anisotropic flagellar controls to regulate swimming symmetry and cell steering" was retracted in 2021. Reasons: unreliable data; unreliable results or conclusions.

## RESULTS

### The human sperm flagellum rotates the cell to beat equally on all sides in 3D

The rapid movement of human sperm flagella was recorded with high spatiotemporal resolution in 3D, as described in Materials and Methods. Two groups of free-swimming spermatozoa in low viscosity were investigated: sperm swimming (i) near to and (ii) far from the coverslip (detailed in Materials and Methods). Figure 2 (A and C) shows, respectively, the flagellar beating of a spermatozoon swimming near and far from coverslip relative to the laboratory fixed frame of reference. The flagellar beat is characterized by a distinctive rolling motion around the swimming direction. The combined rolling and translation motion of the sperm flagellum leads to helical trajectories of the mid-flagellar point with conserved chirality (red traces in Fig. 2, A and C. Spermatozoa displayed bidirectional rolling around their rolling axis; although all free-swimming cells (28 cells) rolled counterclockwise when viewed from the anterior end (arrows in Fig. 2, B and D), only two cells were observed to roll in the clockwise direction (nonprogressive cells due to obstacles in their path) (see Supplementary Text and fig. S4). All spermatozoa (30 cells) were observed to move similarly to a precessing spinning top, in which head spinning around the sperm’s longitudinal axis, referred to as ω_spin_, occurs at the same time as, and independently of, the flagellar rolling around the swimming axis, referred to as ω_roll_, as shown in movie S2. No correlation is observed between “head spinning” and “flagellar rolling” (Fig. 7D); thus, these terms are differentiated here (Fig. 1).

The article "Human sperm uses asymmetric and anisotropic flagellar controls to regulate swimming symmetry and cell steering" was retracted in 2021. Reasons: unreliable data; unreliable results or conclusions.

**Fig. 2:** 3D flagellar beating of human spermatozoa. Sperm swimming near to (**A** and **B**) and far from (**C** and **D**) the coverslip: (A and C) flagellar waveform relative to the laboratory fixed frame of reference (*x*, *y*, *z*) and (B and D) relative to the comoving frame of reference (*x_c_*, *y_c_*, *z_c_*) (see Materials and Methods). In (A) to (D), color progression of the waveform through the flagellar rolling cycle is indicated by the cyclic color map inset, with periods of 474 ms for (A) and (B) and 285 ms for (C) and (D). The red curves depict the trajectory of the mid-flagellar point, indicated by the red plane cross section in (B) and (D). Light gray areas in (A) to (D) show the flagellar projection highlighting the shadow of the wave envelope in each plane. Note that 2D microscopy can only capture the planar *xy* projection depicted. The flagellum rotates around the mean swimming axis, i.e., the rolling axis, depicted by the black straight line in (B) and (D) with the arrow indicating the rolling direction. (B) and (D) show highly symmetric beating in both planar (*xy*) and out-of-plane direction (*z*), see also movies S2 and S3 showing (A) and (B). (A and B) and (C and D) show results for sperm sp6 and sp23, respectively, as described in Materials and Methods.

Figure 2 (B and D) show the flagellar beat, as seen from the comoving frame of reference, i.e., at the view point moving with the spermatozoon but not rolling around its swimming axis (see Materials and Methods). This unveils that the flagellar beat is highly symmetric in both planar (*xy*) and out-of-plane (*z*) directions, beating equally on all sides in 3D (compare the light gray shadows in both *xy* and *zx* planes). The projection of the mid-flagellar trajectory (red curves in Fig. 2, B and D, known as flagelloids (*39*), displayed a bewildering array of geometrical patterns, from rotating star shapes to triangles, squares, and looping patterns with polar symmetry (fig. S4), in agreement with previous reports (*12*, *39*–*41*). Irregular flagelloid patterns, as shown in Fig. 2D for a sperm swimming away from the coverslip, are also observed for sperm swimming near to the coverslip (see, for example, sperm sp1 to sp4 and sp12 to sp18 in fig. S4). This variability in patterns may be induced by phase-lag incongruences between the planar and out-of-plane components of the beat for each cell (Fig. 3), which are magnified in the time scale of the rolling motion. Hence, flagelloid patterns are not a distinguishing feature of cells swimming near to and far from the coverslip. The 3D wave amplitude is characterized by a symmetric bullet-shaped envelope (Fig. 2, B and D and fig. S1), in contrast with the conical helix (similar to a widening corkscrew), which is often postulated (*9*, *10*, *42*). Spermatozoa swimming far from the coverslip displayed a more symmetric waveform envelope than the cells swimming near to the coverslip (fig. S1). The nearby coverslip is thus a weak source of asymmetry to the beat. Furthermore, the flagellar waveform oscillates between purely planar and weakly nonplanar shape at each instant, in agreement with earlier observations (*12*). Spermatozoa swimming near the coverslip displayed a conserved angle of attack of −7°, with the average orientation of the sperm flagellum directed toward the coverslip, as detailed in Supplementary Text and fig. S1.

The article "Human sperm uses asymmetric and anisotropic flagellar controls to regulate swimming symmetry and cell steering" was retracted in 2021. Reasons: unreliable data; unreliable results or conclusions.

**Fig. 3:** Human sperm beats anisotropically and asymmetrically in 3D. (**A** to **D**) The comoving frame of reference (*x_c_*, *y_c_*, *z_c_*) for spermatozoon sp6 in Fig. 2 (A and B) with rolling axis upright (black line) and arrow showing the rolling direction in (A) and (B). (**E** to **H**) The comoving-rolling frame of reference (*x_cr_*, *y_cr_*, *z_cr_*) showing waveform in absence of rotation around the rolling axis (black line) in (E) and (F). Movies S3, S4, and S5 show fixed, comoving, and comoving-rolling frames of reference. (E) Three beating planes are introduced as follows: “*b* plane” (blue) captures the *xy* planar projection, “*z* plane” (red) captures the out-of-plane motion, and “rolling plane” (green) is the plane perpendicular to the rolling axis. (B and F) Principal components analysis (PCA) reconstruction using the first two PCA modes. Inset shows the cyclic color map for (A), (B), (E), and (F) with a period of 474 ms; light-gray areas show flagellar projections highlighting the wave envelope in each plane. (C) and (G) show the time evolution of the first PCA mode (blue) and second PCA mode (orange) for different views [left and right plots in (C) and (G)]. (D and H) Fourier analysis of the waveform. For both (D) and (H): left plot, static (black) and dynamic (red) Fourier modes; middle plot, Fourier reconstruction of the waveform using a superposition of the static mode (black) and dynamic mode (red); and right plot, original data. Frame of references, PCA, and Fourier analyses are detailed in Materials and Methods.

The article "Human sperm uses asymmetric and anisotropic flagellar controls to regulate swimming symmetry and cell steering" was retracted in 2021. Reasons: unreliable data; unreliable results or conclusions.

### The human sperm beats anisotropically and asymmetrically

Figure 3 contrasts the flagellar beat, as seen from the comoving frame of reference (top row) and the comoving-rolling frame of reference (bottom row) (see Materials and Methods). Figure 3E shows the true nature of the flagellar beat, as seen from the spermatozoon’s view point, unbiased by any swimming and rolling motions (fig. S5 and movie S5). The comoving-rolling frame of reference (Fig. 3E) reveals that the flagellar beat is anisotropic, i.e., the wave characteristics in each transversal direction (perpendicular beating planes), denoted by “*b* plane” (blue plane) and “*z* plane” (red plane), differ markedly. Compare the light gray areas at the blue and red planes in Fig. 3E. The beating is highly asymmetric at the *b* plane and characterized by a distinctive broken left-right symmetry resembling a “C” shape (Fig. 3E blue plane). This is in contrast with the remarkably symmetric patterns observed at the comoving frame of reference in Fig. 3A.

Principal components analysis (PCA) of the 3D waveform (detailed in Materials and Methods) allows the decomposition of the beat in terms of a few “principal shape modes,” referred here as PCA modes. The 3D waveform can be reconstructed with good accuracy with only two shape modes, as depicted in Fig. 3 (B and F) and figs. S6 and S7. Figure 3C reveals that the first two PCA modes are identical in shape, up to a 90° rotation (compare the blue and orange surfaces), thus capturing the streamlined helical shape caused by the sperm rolling (see movie S4). In Fig. 3G, however, the intrinsic asymmetric C shape is fully detected by the first PCA mode alone (blue surface). The second PCA mode in Fig. 3G (orange surface) contributes with small deviations perpendicular to the first PCA mode (blue surface), indicating that the waveform may be decomposed into two independent, transversal, beating directions, thus anisotropic in nature.

Fourier analysis of the beat allows the reconstruction of the flagellar movement using only two Fourier modes in Fig. 3 (D and H) (see Materials and Methods for details). Briefly, each generic signal of the beat can be approximated by a simple sum of two functions, *f_r_*(*s*, *t*) ≈ *f*^0^(*s*) + ∣*f*^1^(*s*)∣ sin (ω*t* + ϕ(*s*)). The first term *f*^0^(*s*) is time independent, referred to as the “static mode,” and captures the averaged asymmetry of the signal along the arc length *s* of the flagellum. The second function is a sinusoidal traveling wave, referred to as the “dynamic mode,” oscillating with frequency ω captured by the first peak of the signal’s power spectrum. The amplitude and phase modulations of the traveling wave along the flagellum are, respectively, ∣*f*^1^(*s*)∣ and ϕ(*s*) = arg (*f*^1^(*s*)) (see Materials and Methods). The phase thus carries information about the traveling wave characteristics, for example, if the phase ϕ(*s*) does not vary along *s*, then the signal is not a traveling wave but rather a standing wave.

The article "Human sperm uses asymmetric and anisotropic flagellar controls to regulate swimming symmetry and cell steering" was retracted in 2021. Reasons: unreliable data; unreliable results or conclusions.

Hence, the static mode captures any shape incongruence of the waveform; thus, the black straight line in Fig. 3D reflects the beating symmetry in both *xy* and *xz* planes in comoving frame. In contrast, in the comoving-rolling frame in Fig. 3H, the static mode (black curve) is characterized by a large asymmetric amplitude, resembling an inverted C. The dynamic mode in the comoving frame (red curves) in Fig. 3D has a large amplitude and is highly symmetric in both *xy* and *xz* planes due to sperm rolling. In contrast, the dynamical mode (red curves) in the comoving-rolling frame (Fig. 3H) has a reduced waveform amplitude and, instead, a preferential direction of motion. The Fourier reconstruction of the waveform is given by combined action (sum) of the static and dynamic modes, depicted by the middle plots in Fig. 3 (D and H), which agrees well with the original observations (right plots in Fig. 3, D and H).

### The human sperm uses two coactive transversal controls: An asymmetric traveling wave and a pulsating standing wave

Figure 4 shows the Fourier analysis of the 3D flagellar beat across the free-swimming sperm population for a total of 28 spermatozoa (20 cells near to and 8 cells far from the coverslip, as described in Materials and Methods). At the comoving frame (Fig. 4, A to C), the amplitudes of the static mode in both directions, (*y_c_*, *z_c_*), are very small (top row of Fig. 4, B and C) due to the beating symmetry. Moreover, the amplitude (middle row) and phase (bottom row) of (*y_c_*, *z_c_*) dynamical modes in Fig. 4 (B and C) are analogous, capturing the transversal symmetry and thus beating isotropy at this frame of reference due to the sperm rolling around the swimming axis (compare figs. S16 and S17). The traveling wave characteristics of both *y_c_* and *z_c_* coordinates (calculated from phase in the bottom row of Fig. 4, B and C; see Materials and Methods) are similar across the free-swimming population, averaging a frequency of 4 Hz, a wavelength of 100 μm, and a wave speed of 400 μm/s. The sperm rolling frequency ω_roll_ also averages 4 Hz across the population, as expected from the periodicity of (*y_c_*, *z_c_*) in this frame of reference.

**Fig. 4:** The 3D flagellar beating is a transverse superposition of a traveling wave and a standing wave. Fourier analysis of each transverse plane across the free-swimming sperm population for a total of 28 spermatozoa: 20 cells near to the coverslip and 8 cells far from the coverslip, with heights between 0 and 85 μm, as detailed in Materials and Methods. (**A** and **D**) The comoving and comoving-rolling frame of references, respectively, for the spermatozoon sp6 depicted in Fig. 3. (**B** and **C**) Columns, for the comoving frame coordinates (*y_c_*, *z_c_*); (**E** and **F**) Columns, for the comoving-rolling frame coordinates, (*y_cr_*, *z_cr_*), denoted, respectively, by *b* plane (E) and *z* plane (F). In (B), (C), (E), and (F), top and middle rows show the amplitude of the static and dynamic modes rescaled by 1.6 μm, respectively, as a function of arc length. The bottom row shows the phase of the dynamical mode as a function of arc length. Black curves depict averages in the free-swimming sperm population. The transformations between referential frames and Fourier analysis are detailed in Materials and Methods.

The article "Human sperm uses asymmetric and anisotropic flagellar controls to regulate swimming symmetry and cell steering" was retracted in 2021. Reasons: unreliable data; unreliable results or conclusions.

At the comoving-rolling frame of reference (Fig. 4, D to F), large but distinct static modes in the *b* plane and *z* plane show that the beating has a conserved anisotropy across the free-swimming population (top row of Fig. 4, E and F). The static mode of the *b* plane, *y_cr_*, is highly asymmetric, skewed to positive values (top row of Fig. 4E), while the *z* plane, *z_cr_*, oscillates symmetrically along the arc length in a sinusoidal fashion (top row of Fig. 4F). Both (*y_cr_*, *z_cr_*) static modes are well characterized by a sum of two sine functions by curve fitting with the population mean (black curves in the top row of Fig. 4, E and F), respectively, given by $y_{\mathrm{cr}}^{0}\approx 1.85\;\text{sin}\;(0.07s-0.08)+0.5\;\text{sin}\;(0.15s-3.37)$ and $z_{\mathrm{cr}}^{0}\approx 1-0.65\;\text{sin}\;(0.11s-0.16)-0.07\;\text{sin}\;(0.23s+2.3)$, where *s* is the arc length. The amplitude of the dynamical mode $y_{\mathrm{cr}}^{1}$ at the *b* plane increases until plateauing (middle row of Fig. 4E), while the dynamical mode $z_{\mathrm{cr}}^{1}$ at the *z* plane is nonmonotonic along the arc length (middle row of Fig. 4F). The latter is due to the fact that the mid-flagellum is the reference point capturing the flagellar rolling in the comoving-rolling frame of reference (see Materials and Methods); therefore, by definition, *z_cr_* = 0 at this point in arc length.

The phase of the dynamical mode of *y_cr_*, $\text{arg}\;(y_{\mathrm{cr}}^{1})$, decreases along arc length (bottom row of Fig. 4E). Phase differences along flagellar length are expected for traveling waves; the rate of decay of the phase captures the wave speed (see Materials and Methods). Thus, the wave speed of *y_cr_* is weakly nonlinear along the arc length (see also fig. S18). Traveling wave characteristics of *y_cr_* (*b* plane) averaged a frequency of ω*_y_cr__* = 8 Hz across the free-swimming population, a wavelength of 145 μm, and a wave speed of 1120 μm/s. On the other hand, *z_cr_* (*z* plane) oscillates with an average frequency of ω*_z_cr__* = 6 Hz, a wavelength of 1526 μm, and a wave speed of 5174 μm/s across the free-swimming population. These high values of wave speed/wavelength are due to the almost constant arc length profile of the phase $\text{arg}\;(z_{\mathrm{cr}}^{1})$ along the flagellum (bottom row of Fig. 4F and fig. S13). Small changes in phase across long flagellar distances require very rapid wave propagation speeds. The oscillations of *z* plane thus effectively behave as a standing wave pulsating in time. These pulsating standing waves are equally apparent in the kymographs of *z_cr_* in fig. S19.

The article "Human sperm uses asymmetric and anisotropic flagellar controls to regulate swimming symmetry and cell steering" was retracted in 2021. Reasons: unreliable data; unreliable results or conclusions.

The flagellar beat thus uses two coactive anisotropic transversal controls, not too dissimilar from electromagnetic traveling waves. Here, however, each transversal wave (*y_cr_*, *z_cr_*) is a sum of a static and a dynamical mode: an asymmetric traveling wave along the *b* plane (blue) and a symmetric standing wave in the *z* plane (red) (Fig. 4D and figs. S18 and S19).

### The coverslip’s solid boundary affects the flagellar beat anisotropically

The presence of the nearby coverslip decreases the amplitude of the wave propagation in 3D (Fig. 5 and figs. S1, S12, and S13), potentially due to the hydrodynamic interactions between the flagellum and the solid boundary of the coverslip (*6*, *43*). In the comoving frame of reference (Fig. 5, A and B), the amplitude of both the (*y_c_*, *z_c_*) dynamical modes are reduced toward the end piece for sperm near to the coverslip (middle plots), while the static modes remained unchanged (top plots). The dynamical mode of *z_c_* is only slightly smaller than *y_c_* (blue curves) in the middle plots of Fig. 5 (A and B). This is in contrast to the symmetric, unchanged, profiles of both (*y_c_*, *z_c_*) dynamical modes for spermatozoa found away from the boundary (red curves in the middle plots of Fig. 5, A and B). At the comoving-rolling frame of reference in Fig. 5 (C and D), however, the influence of the coverslip is distinctively anisotropic, as it only affects one beating plane, the *b* plane (*y_cr_*; Fig. 5C). The coverslip influences both static and dynamic modes of *y_cr_* in Fig. 5C (top/middle). In contrast, the *z* plane *z_cr_* remains unchanged for cells swimming near to the coverslip (see Fig. 5D, top/middle). In all cases, the phase is weakly perturbed by the solid boundary (bottom row of Fig. 5, A to D).

The article "Human sperm uses asymmetric and anisotropic flagellar controls to regulate swimming symmetry and cell steering" was retracted in 2021. Reasons: unreliable data; unreliable results or conclusions.

**Fig. 5:** Hydrodynamic modulation of the beat by the coverslip and the logarithmic flagellar helix are anisotropic. Each column (**A** to **D**), from top to bottom, respectively, the averages for spermatozoa swimming near to (blue; 20 cells) and far from (red; 8 cells) the coverslip of the static and dynamic modes and phase of *y_c_* (A), *z_c_* (B), *y_cr_* (C), and *z_cr_* (D) from Fig. 4. Sperm swimming far from the coverslip ranged their heights between 20 and 85 μm, as detailed in Materials and Methods. The static mode is a logarithmic-like helix that dictates the sperm rolling direction in (E) to (H). (**E**) The averaged static mode of the coordinates $y_{\mathrm{cr}}^{0}$ and $z_{\mathrm{cr}}^{0}$ across the population, shown in the top row of Fig. 4 (C and D) by the black curves, defines a right-handed helix in 3D (black curve), denoted by ***h***(*s*). The helix projection at the rolling plane (green plane) is an asymmetric, counterclockwise spiral (gray curve). The *b* plane and *z* plane are shown, respectively, by the blue and red planes. Arrows depict the Frenet basis (normal and binormal vectors) showing that the helix is right handed (see Materials and Methods). The dashed straight line is the rolling axis; (**F**) radius of the spiral *r* in polar coordinates (*r*, α) as a function of arclength *s* (black curve); (**H**) radius squared of the spiral, *r*^2^, in function the polar angle α (black curve), with blue squares showing the linear regression before and after the maximum at α = 0, denoted by *r*_max_. The red curve and blue squares in (F) show, respectively, the Gaussian fit and the linear regression, as in (H), but only for the first half before *r*_max_ ; (**G**) pitch of the helix, *p*(*s*), as a function of arc length *s* (black curve) and its exponential fit (red curve), see main text for details.

### The shape of the static mode is reminiscent of a logarithmic helix and governs the sperm rolling bidirectionality

The shape of the static mode in the comoving-rolling frame is conserved across all the sperm population (for both free-swimming and nonprogressive cells) and defines an off-centered, right-handed helix in 3D, denoted by **h**(*s*) and shown by the black curve in Fig. 5E. The projection of the helix at the rolling plane (green plane) is a counterclockwise spiral that lacks polar symmetry, i.e., it is skewed to one side (gray projection in Fig. 5E). The helix “unfolds” the spiral along the rolling axis, which is given by the intersection of the blue and red planes in Fig. 5E. The radius of the spiral *r* is a nonmonotonic function of both arc length *s* and the polar angle α in Fig. 5 (F and H). The slope of *r*^2^, before and after *r* = *r*_max_ (Fig. 5H), is approximately constant and symmetric, as shown by the linear square markers in Fig. 5H. The spiral around *r*_max_ is thus well approximated by a superposition of two Fermat spirals, with positive and negative slopes, respectively, before and after the maximum value, with *r*^2^ ≈ ± *a*^2^α and *a*^2^ = 16.89. The spiral radius, however, has a Gaussian distribution around *r*_max_ reflecting its nonmonotonicity, with *r*(*s*) = 2.2 exp [− ((*s* − 28.12)/16.68)^2^], depicted by the red curve in Fig. 5F. The spiral of the static mode is thus reminiscent of logarithmic spirals that are frequently found in nature, with *r* = *a e*^*b*α^ and generic constants *a*, *b* ≠ 0. However, here, the spiral radius varies nonmonotonically, increasing/decreasing at a higher rate than logarithmic spirals elsewhere in nature.

The article "Human sperm uses asymmetric and anisotropic flagellar controls to regulate swimming symmetry and cell steering" was retracted in 2021. Reasons: unreliable data; unreliable results or conclusions.

The right-handed, logarithmic-like helix in Fig. 5E can be expressed in terms of its radius *r*(*s*) and pitch *p*(*s*), as **h**(*s*) = (*h_x_*, *h_y_*, *h_z_*) ≈ (*s*, *r* cos (*sl*), *r* sin (*sl*)) via the wave number *l*(*s*) = (*r*^2^ + *p*^2^)^−1/2^. The pitch *p*(*s*) (Fig. 5G) decays exponentially along the flagellar length, according to *p*(*s*) = 1651 exp (−0.53*s*) + 84 exp (−0.03*s*). Any sign change in either *h_y_* or *h_z_* causes the handedness of the spiral to switch to a clockwise spiral, generating instead a left-handed helix. All free-swimming spermatozoa generated counterclockwise spirals and, thus, right-handed helices for their static modes, as in Fig. 5E. Only two spermatozoa were observed with clockwise spirals, although with shapes identical to Fig. 5E under sign change *h_z_* → −*h_z_*. Incidentally, these two cells (spermatozoa sp29 and sp30 in Materials and Methods and Supplementary Text) were prevented from swimming forward by obstacles in their path, although were still able to rotate around their rolling axis (see movie S6), similar to experiments performed by Ishijima *et al.* (*44*). In all cases, the handedness of the spiral correlated with the sperm rolling direction as follows: counterclockwise spiral for clockwise rolling (when seen from the posterior end) and clockwise spirals for counterclockwise rolling (also further discussed in Supplementary Text).

### 3D traveling waves of curvature and waveform perversion

The 3D curvature κ and torsion τ of the flagellum centerline were measured directly from the flagellar waveform. The curvature captures the actual “bending” of the flagellum in 3D, while the torsion measures the “three dimensionality” of the centerline via its out-of-plane turns in space (see Materials and Methods). Figure 6 (A and B) shows a complex train of traveling waves, as the flagellum rotates around its rolling axis. Bending waves travel linearly along the flagellum (black slope in Fig. 6D) with a nonmonotonic amplitude along the arc length, characterized by an abrupt increase in the midpiece and the distal regions (see static mode κ^0^ in Fig. 6H). The waveform torsion is characterized by sharp traveling turns along the arc length (Fig. 6, B and C) with coexisting positive and negative turns in the same instant (see blue and yellow ribbons in Fig. 6C or, equally, the propagating yellow and blue peaks in Fig. 6E). The helical shape of the flagellum centerline undergoes a “perversion” phenomenon by which sections of opposite chirality (handedness) along the flagellum coexist (*12*, *45*, *46*). Here, however, the flagellar sections of opposite chirality travel during the beat (Fig. 6, C and E). The traveling waves of torsion, or rather perversion, propagate with the same speed as the wave of curvature (see linear decay in the bottom row of Fig. 6, H and I), however, with the manifestation of phase jumps in torsion (sudden changes from blue to yellow in Fig. 6E) and time delays between the wave propagation of κ and τ.

The article "Human sperm uses asymmetric and anisotropic flagellar controls to regulate swimming symmetry and cell steering" was retracted in 2021. Reasons: unreliable data; unreliable results or conclusions.

**Fig. 6:** Helical waves of flagellar perversion. (**A**) Typical flagellar bending around the rolling axis (black line) with ribbon’s color showing the torsion intensity as in (C). (**B**) Time series of the 3D waveform with ribbon’s color showing the magnitude in curvature κ in units of μm^−1^. (**C**) Torsional waves in the absence of bending deformation with ribbon colors showing the torsion τ in units of μm^−1^. All twisted ribbons in (A) to (C) show the torsional angle of rotation along the flagellum (see Materials and Methods). (**D** to **G**) Kymographs of the curvature κ, torsion τ, spiral’s curvature κ*_s_* (projection in the rolling plane), and the chirality ψ in radians as a function of arc length *s* and time *t* (see Materials and Methods). Overlaid black line indicates that the speed of propagation in (D) to (G) is the same. The dashed lines in (D) to (G) show the time duration depicted in (B) and (C). (**H** and **I**) Top to bottom is as follows: amplitude of the static and dynamic modes and phase, respectively, for (H) column the curvature κ and (I) column the absolute torsion ∣τ∣, with black curves depicting averages across all free-swimming spermatozoa (see Materials and Methods). (D to I) Curvature and torsion are in units of μm^−1^. (A) to (G) show results for sperm sp8 (see Materials and Methods). The waveform parameters and Fourier analysis are detailed in Materials and Methods.

The article "Human sperm uses asymmetric and anisotropic flagellar controls to regulate swimming symmetry and cell steering" was retracted in 2021. Reasons: unreliable data; unreliable results or conclusions.

The curvature of the spiral κ*_s_* in Fig. 6F, defined as the waveform projection at the rolling plane (see Materials and Methods), is a linear propagating wave of peaks, similar to the torsional waves (compare the straight lines in Fig. 6, E and F). This is due to the formation of sharp kinks in this projection. Incidentally, κ*_s_* propagates similarly to κ (compare Fig. 6, D and F). Large torsion occurs when either κ or rather κ*_s_* approaches zero, as the centerline torsion scales with $\tau \propto 1/\kappa_{s}^{2}$. That is, when the curvature is small, the torsion is large if the out-of-plane component of the waveform is nonzero, leading to the observed phase lag between curvature and torsion in Fig. 6 (D and E). The flagellar perversion is propagated with wave characteristics similar to the curvature (compare Fig. 6, G and D). Nevertheless, the local chirality is not conserved, as indicated by the change in handedness (sign changes) in Fig. 6G and fig. S23.

The static and dynamic modes of κ and ∣τ∣ across the free-swimming population are shown in Fig. 6 (H and I). The curvature static mode (top row of Fig. 6H) increases nonmonotonically and has two local maxima. The absolute torsion static mode (top row of Fig. 6I) also has a rapid increase in the midpiece from which the amplitude decays. The curvature dynamic mode (middle row of Fig. 6H) increases linearly before reaching a maximum at the distal end, while the absolute torsion dynamic mode (middle row of Fig. 6I) is parabolically distributed along the length. Curvature and torsion average similar wave characteristics, with a frequency of 14 Hz (16 Hz), a wavelength of 38 μm (31 μm), and a wave speed of 415 μm/s (452 μm/s) for the curvature (torsion), as shown in the bottom row of Fig. 6 (H and I). Hence, the strong correlation in Fig. 7A between the beating frequency, defined by the first peak of the Fourier spectrum of the curvature ω_κ_ (as depicted in Fig. 7F), and the torsion’s frequency ω_τ_. Figure 7 (B and C) shows, respectively, a strong correlation between ω_τ_ and the head spinning frequency ω_spin_ and between ω_κ_ and the flagellar rolling frequency ω_roll_, indicative of separate controls for the head spinning and flagellar rolling. No correlation is observed between the head spinning and flagellar rolling in Fig. 7D, as expected from the asymmetry of the beat in Fig. 5E and detailed in Discussion.

**Fig. 7:** Flagellar rolling and head spinning, hydrodynamic modulation, and 2D microscope projections. (**A**) Correlation between the beating frequency, defined by the first peak of the Fourier spectrum of the 3D curvature [red curve in (F)], ω_κ_, and the torsion’s frequency, ω_τ_. (**B**) Strong correlations between torsion ω_τ_ and the head spinning frequency ω_spin_ and (**C**) between curvature ω_κ_ and flagellar rolling frequency ω_roll_. (**D**) No correlation exists between head spinning, ω_spin_, and flagellar rolling frequency around the swimming axis, ω_roll_. (**E**) From top to bottom, respectively, the averages across the population of the static and dynamic modes and phase of the curvature κ, for the sperm near to (blue; 20 cells) and far from (red; 8 cells) the coverslip. Sperm swimming far from the coverslip ranged their heights between 20 and 85 μm, as detailed in Materials and Methods. (**F** and **G**) 2D microscopy fails to capture beating asymmetry: (F) Typical Fourier spectrum of the 3D curvature (red) and the 2D curvature κ_2D_ (black), obtained by projecting the 3D waveform in the *xy* plane (gray curves in Fig. 2, B and D and Materials and Methods). The first peak in κ (red) defines the beating frequency ω_κ_. κ_2D_ is characterized instead by two frequency peaks (black markers), denoted by $\omega_{\kappa 2D}^{1,2}$, while zeroth mode (static mode) is zero. (G) No correlation exist between the first frequency peak of the 2D curvature $\omega_{\kappa 2D}^{1}$ and the head spinning ω_spin_.

The article "Human sperm uses asymmetric and anisotropic flagellar controls to regulate swimming symmetry and cell steering" was retracted in 2021. Reasons: unreliable data; unreliable results or conclusions.

The proximity to the coverslip modulates the beat in 3D by reducing the amplitude of both static and dynamic modes of the curvature toward the distal end (blue curves at top and middle rows of Fig. 7E and fig. S14), similar to *y_cr_* in Fig. 5C. The phase of κ is weakly affected by the coverslip (as shown in the bottom row of Fig. 7E): Spermatozoa swimming near to (far from) the coverslip were observed to beat slightly faster (slower), with an average frequency of 15 Hz (11 Hz), a wavelength of 35 μm (42 μm), and a wave speed of 429 μm/s (392 μm/s).

### 2D microscopy fails to capture beating asymmetry and anisotropy

Traditional 2D microscopy captures planar projections of the 3D excursions of the flagellar beat. 2D projections were obtained directly from the 3D waveform, as depicted by the light gray curves in the *xy* plane in Fig. 2A, from which the 2D curvature κ_2D_ is calculated (see Materials and Methods). The static mode (zeroth Fourier mode) of the 2D curvature κ_2D_ is negligible (black curve in Fig. 7F and fig. S15). No intrinsic waveform asymmetry can be detected in 2D. The frequency spectrum is characterized instead by two frequency peaks (black markers in Fig. 7F) rather than a single main frequency peak observed for the 3D curvature κ (red curve in Fig. 7F and figs. S24 and S25). The first frequency peak of κ_2D_, denoted by $\omega_{\kappa 2D}^{1}$, postulated to be related with the head spinning frequency, ω_spin_, shows no correlation in Fig. 7G. The first frequency peak $\omega_{\kappa 2D}^{1}$ correlates instead with the flagellar rolling frequency (fig. S2), as expected from the 2D projection of the comoving frame of reference (Fig. 2B). The second frequency peak of the 2D curvature spectrum, $\omega_{\kappa 2D}^{2}$, correlates strongly with the beating frequency ω_κ_ (*R* =0.82 in fig. S2), although κ_2D_ underestimates wave parameters. κ_2D_ also displays a nonexistent linear increasing amplitude due to the absence of the static mode (fig. S15), which have been the basis of numerous waveform hypotheses (*2*, *6*, *15*, *47*), as discussed in Supplementary Text.

The article "Human sperm uses asymmetric and anisotropic flagellar controls to regulate swimming symmetry and cell steering" was retracted in 2021. Reasons: unreliable data; unreliable results or conclusions.

## DISCUSSION

We used high-precision 3D video microscopy to resolve the rapid movement of the human flagellum in 3D. This allowed the description of the flagellar waveform relative to both the comoving and rolling frame of reference of the sperm flagellum. This unveiled the true nature of the waveform unbiased by the sperm swimming and rolling motions. The human sperm flagellum beating, postulated be symmetric, is skewed with a broken left-right symmetry in one plane (*b* plane), with a small but symmetric out-of-plane component (*z* plane). The rolling motion enables spermatozoa to swim in a straight trajectory despite its biased waveform. This is achieved via a coordinated 360° rotation of asymmetric one-sided bends around the rolling axis, driving symmetric excursions of the flagellum on all sides in 3D (Figs. 1 and 2, B and D). The rolling-of-asymmetric-bend mechanism induces an optical illusion if seen with traditional 2D microscopy, i.e., the flagellar beating appears to have symmetric side-to-side movement for free-swimming and rolling spermatozoa (*4*, *5*, *7*, *8*, *47*).This rendered the intrinsic beating asymmetry of the human sperm invisible thus far. Similar rolling-of-asymmetric-bend mechanism has also been reported for murine spermatozoa (*37*). In this case, however, the flagellum induces a rapid 180° switch from one side to the other, in contrast with the gradual 360° rolling of human sperm observed here.

The flagellar movement in 3D is a combination of a planar and out-of-plane motion captured, respectively, by the *b* and *z* plane components (Fig. 4D). The flagellum motion in each plane is a sum of two independent shape modes: a static mode whose shape does not change in time and a dynamic mode that oscillates in time (see Materials and Methods). The waveform of each beating plane shares antagonistic properties: The static mode of the *b* plane is asymmetric along the flagellum, while the *z* plane is symmetric (Fig. 4, E and F). Likewise, the dynamic mode of the *b* plane is a traveling wave, while the *z* plane pulsates as a standing wave (Fig. 4, E and F). The 3D flagellar beating is thus anisotropic and given by the coaction of two transversal controls that regulate an asymmetric traveling wave and a pulsating wave along the flagellum. The standing wave in the *z* plane critically modulates the three dimensionality of the beat (fig. S1), thus vital for the spontaneous coordination of sperm rolling (Fig. 2, B and D and fig. S4). No rolling motion of the spermatozoa may emerge without the out-of-plane component of the beat. Thus, if the waveform amplitude of the *z* plane is negligible, then the spermatozoa would potentially only swim in circles, driven by the asymmetric one-sided stroke of the *b* plane. Likewise, observation of circular swimming trajectories in human sperm may be associated with distinct flagellar controls of the *z* plane (*4*, *5*, *47*, *48*).

The article "Human sperm uses asymmetric and anisotropic flagellar controls to regulate swimming symmetry and cell steering" was retracted in 2021. Reasons: unreliable data; unreliable results or conclusions.

The shape of the static mode defines a skewed, right-handed helix whose projection in the rolling-plane is a counterclockwise spiral reminiscent of logarithmic spirals found in nature (Fig. 5E). In general, the helix is ambidextrous, defining a clockwise or counterclockwise spiral (see Materials and Methods). The spiral shape of the static mode works as a “wave guide” for the propagation of the dynamic mode (Fig. 4, E and F). As a result, the rolling direction is dictated by the spiral’s handedness, given that traveling waves always propagate from the proximal to the distal direction along the flagellum. The helical flagellum thus rotates around the rolling axis in the opposite direction of the spiral’s traveling wave due to the total balance of momentum of a free-swimming sperm. Human spermatozoa with a counterclockwise spiral (right-handed helix) rolled clockwise (when seen from the posterior end), while clockwise spirals (left-handed helix) rolled counterclockwise (see Supplementary Text and fig. S4).

The waveform torsion is characterized by rapid turns in both directions with phase jumps and time delays between distant parts of the flagellum (Fig. 6). This unveiled a new waveform perversion phenomenon manifested via kinks connecting helices of opposite chirality along the flagellum (*45*). Traveling waves of perversion induce the lack of local persistent chirality, as previously observed for malaria flagella (*46*) and human spermatozoa (*12*) and shown here with a finer resolution (Fig. 6G and fig. S23). Paradoxically, sperm swimming trajectories define helices of conserved handedness (*12*–*14*, *37*), as depicted by the red curve in Fig. 2A and movie S2. According to the current paradigm, there should be a connection between the handedness of the waveform and the handedness of the helical path that it generates. This connection, however, is based on the assumption of symmetry, where the waveform is often idealized as a conical helix in 3D (*9*–*11*), similar to a widening corkscrew. The inherent asymmetries of the flagellar beat, however, disconnect the local handedness of the waveform from the handedness of the helical trajectories (*12*, *46*); the head spinning and flagellar rolling are not correlated (Fig. 7D). Instead, they appear to be independently controlled: Torsional waves are strongly correlated with head spinning (Fig. 7B), while curvature waves are strongly correlated with flagellar rolling (Fig. 7C). This suggests that traveling waves of torsion induce the sperm rotation along its longitudinal axis and drive head spinning. On the other hand, the flagellar rolling around the swimming axis, responsible for the conserved chirality of the helical trajectory, is dictated by large one-sided curvature waves. The handedness of the spiral static mode is dominant and dictates the sperm rolling direction (Figs. 4, E and F and 5E). This creates the effect of a precessing spinning top, in which the spinning head “drills” into the fluid, and, at the same time, the sperm flagellum rolls around the swimming axis (Fig. 1 and movie S2). This thus reconciles the previously unexplained disconnection between observations of variable chirality of the waveform and the conserved chirality of its helical path.

The article "Human sperm uses asymmetric and anisotropic flagellar controls to regulate swimming symmetry and cell steering" was retracted in 2021. Reasons: unreliable data; unreliable results or conclusions.

Human spermatozoa may achieve high levels of control of the flagellar helical handedness and subsequent rolling motion, without requiring complex regulatory mechanisms. This could be achieved, for example, by simply shaping the static mode with a stable asymmetric binding of molecular motors on one side of the flagellum (*25*). Sign changes of any coordinate component of the spiral can switch the handedness of the flagellar helix. Likewise, flagellar buckling may also modify the spiral’s handedness and the sperm rolling direction, for example, when spermatozoa are prevented from swimming freely due to obstacles, although are still free to rotate around their rolling axes (movie S6) (*44*). This potentially conciliates contradictory observations showing unidirectional, bidirectional, and even intermittent directionality of rolling in human spermatozoa (see Supplementary Text) (*12*–*14*, *37*, *44*).

### Molecular and structural origin of beating asymmetry and anisotropy

The logarithmic helix of the static mode entails that internal forces along the flagellum are nonuniform, asymmetric, and helically distributed (Fig. 5E), in contrast with the circular arcs in *Chlamydomonas* mutants (*29*). Our observations are consistent with reports showing a hierarchy of distinct asymmetries in flagellar systems, from asymmetric distribution and activity of molecular motors (*25*, *31*, *32*) to asymmetric bending in hamster spermatozoa (*37*), asymmetric static modes in *Chlamydomonas* (*23*, *27*), atypical centriole (*33*), and an ever growing number of asymmetric regulatory complexes (*10*, *27*, *29*, *34*, *35*) in addition to other unknown biases from less well-studied motor proteins (*36*). While the exact molecular mechanism underlying the observed asymmetric static shape is still unknown (*23*, *27*), our results show that, together with murine spermatozoa (*37*) and *Chlamydomonas* flagellum (*23*), the human sperm flagellum is part of the asymmetric beating–flagellated microorganisms that exhibit an intrinsically asymmetric static mode, reflecting potential universal asymmetries across species.

The article "Human sperm uses asymmetric and anisotropic flagellar controls to regulate swimming symmetry and cell steering" was retracted in 2021. Reasons: unreliable data; unreliable results or conclusions.

The wave amplitude in the *b* plane is much larger than in the *z* plane, which has, instead, a sinusoidal distribution in arc length (top row of Fig. 4, E and F). That is, the waveform is anisotropic, as depicted in Fig. 8A. This may find its origin in the ultrastructural complex reinforcing the axoneme in human sperm (*2*, *20*), represented in Fig. 8 (B and C). Outer dense fibers are connected to the microtubule doublets forming the 9 + 9 + 2 structure. The outer dense fibers 8 and 3, however, are replaced by two diametrically opposite longitudinal columns (LCs) at the principal piece, as shown in Fig. 8C. Thus, this introduces a mechanical anisotropy along the flagellum: It suppresses bending in one direction and facilitates it in the other. The large bending observed in one direction could be facilitated by the “weaker” side of the flagellum so that the *b* plane would lie perpendicular to the LCs (blue double arrow in Fig. 8C). On the other hand, bending could be hindered by the “stronger” side of the flagellum so that the *z* plane would lie parallel to the LCs, as illustrated in Fig. 8C. Coincidently, upon increased hydrodynamic load for sperm swimming near to the coverslip, only modest changes in wave amplitude were observed at the *z* plane (stronger side of the flagellum, see Fig. 5D), while the *b* plane (weaker side) was greatly affected by the nearby surface in Fig. 5C (compare blue and red curves). Last, the sinusoidal shape of the static mode in the *z* plane (top row of Fig. 4F) could also be a manifestation of another flagellar structural effect via, for example, the axonemal counterbend phenomenon (*30*, *49*), in which proximal bending causes the distal end to bend in the opposite direction, resembling the shape of a sine function (top row of Fig. 4F).

The article "Human sperm uses asymmetric and anisotropic flagellar controls to regulate swimming symmetry and cell steering" was retracted in 2021. Reasons: unreliable data; unreliable results or conclusions.

**Fig. 8:** Ultrastructural and molecular origin of the flagellar anisotropy. (**A**) The flagellar beating anisotropy in 3D, as in Fig. 4D, showing the *b* plane and *z* plane. (**B**) Representation of a mammalian sperm flagellum showing the tapering of the reinforcing ultrastructure along the flagellar length (blue), with the axoneme depicted in yellow. (**C**) The cross section of a mammalian sperm flagellum [rectangle in (B)] showing that the 9 + 9 + 2 ultrastructure (*2*) is anisotropic. The 9 + 2 axoneme is surrounded by nine outer dense fibers (gray); however, the outer dense fibers 8 and 3 are replaced by two diagonally opposite LC. The LCs constrain the beating to the weaker side of the flagellum (blue double arrow), thus potentially coaligned with the *b* plane in (A). The reduced amplitudes of the *z* plane (red) in (A) are likely to be suppressed by the stronger side of the flagellum and thus aligned with the plane defined by the LCs (red double arrow). (**D**) Anisotropic bilateral localization of Hv1 proton channels (blue eclipses) compared with the symmetrical, quadrilateral localization of CatSper ion channels (red ellipses) reported by Lishko’s group (*34*), in a flagellar cross section. Dashed circular region (light blue) shows the CatSper channel mostly affected by one of the Hv1 channels in close proximity, which is also located near to one of the LCs, thus affecting molecular motors anisotropically along the stronger side of the flagellum.

Each beating plane is dynamically very distinct: The wave speed of the *z* plane is five times higher, and the wavelength is 10-fold larger than the traveling waves of the *b* plane. Thus, the *z* plane effectively pulsates as standing wave (bottom row of Fig. 4, E and F and fig. S19). This is indicative of independent, although anisotropic, regulatory mechanisms modulating each plane, or else, this would require molecular motors alone to work differently in each beating plane. Furthermore, standing waves in the *z* plane are unlikely to be achieved via molecular motor dynamics alone, as this would require a fast, synchronized motor coordination over long flagellar distances, not yet reported in the literature. Molecular motor self-organization is manifested through time-delayed oscillations along the flagellum (*1*, *18*) which lead to the generation of propagating waves, and therefore is the most likely mechanism to govern the asymmetric traveling waves observed in the *b* plane (Fig. 8A) (*18*, *23*, *25*, *26*).

The standing wave pulsation of the *z* plane indicates the existence of a fast regulator along the flagellum length (Fig. 4F). Ion channels, such as CatSper and Hv1, are docked at the plasma membrane to ensure fast signal transduction along the length of the whole flagellum (Fig. 8D) and are critical for hyperactivation, rheotaxis, and sperm rolling (*10*, *12*, *34*, *35*). Furthermore, species-specific adaptations could also lead to specialized localization of these regulatory complexes. For example, the human sperm flagellum has the largest Hv1 current density due to proton channels of all cell types (*34*, *35*). However, unlike CatSper channels (*10*) which have a symmetrical quadrilateral localization at the flagellar cross section, Hv1 is distributed asymmetrically and unilaterally along the flagellum (*34*) and may be related to the observed pulsation in the *z* plane, as indicated in Fig. 8D.

The article "Human sperm uses asymmetric and anisotropic flagellar controls to regulate swimming symmetry and cell steering" was retracted in 2021. Reasons: unreliable data; unreliable results or conclusions.

The *z* plane modulates the out-of-plane component of the beat (Fig. 8A), its quasi-planarity, and subsequent sperm rolling self-organization. Upon inhibition of Hv1, Miller *et al.* (*34*) demonstrated that the 360° rolling of human sperm was markedly decreased, often leading to partial 180° rolling events, much similar to the motion of murine sperm (*10*, *37*), which indeed lack Hv1 expression (*35*). Hence, given the observed correlation between head spinning and waveform torsion in Fig. 7B, the Hv1 channel may play an important role while regulating the waveform torsion. Furthermore, Miller *et al.* (*34*, *35*) showed that Hv1 may alkalinize a subportion of the axoneme and up-regulate a subset of CatSper channels in close proximity (blue region in Fig. 8D). This would result in a local increase in Ca^2+^, causing the arrest of dyneins and effectively increasing the rigidity, unilaterally, within the flagellum. Most notably, the Hv1 channel likely up-regulates the CatSper located near one of the LCs (dashed blue circle in Fig. 8D), thus potentially only affecting one beating plane, the *z* plane (red double arrow in Fig. 8D). This indicates that, once again, the *z* plane could be coaligned with the plane composed by the LCs, similarly to the localization of the ultrastructural components in Fig. 8C. Thus, the correlation between the position of the LCs and Hv1 channels and the orientation of the *z* plane in Fig. 8D might not be incidental.

Although it is not possible to exactly assert whether the Hv1 channels are responsible or not for the pulsations of the *z* plane observed here, our results show that sperm rolling self-organization cancels out the umbrella of intrinsic asymmetries present at the molecular level, allowing the sperm to swim forward. This resolves the apparent paradox connecting molecular and microscopic observations, by explaining how human sperm can both operate asymmetrically and achieve symmetric side-to-side motion, effectively creating symmetry out of asymmetry. This provides evidence that the sperm flagellum is asymmetrically controlled and anisotropically regulated via fast signal transduction along the flagellar length.

The article "Human sperm uses asymmetric and anisotropic flagellar controls to regulate swimming symmetry and cell steering" was retracted in 2021. Reasons: unreliable data; unreliable results or conclusions.

### 2D observations of symmetric swimming in the context of 3D asymmetric flagellar control

The intrinsic beating asymmetry observed here unearths the current need to reinterpret 2D observations of human sperm swimming. Forward swimming is achieved via the combined action of an asymmetric traveling wave that creates a one-sided swimming stroke and a pulsating standing wave that rolls the sperm to beat equally on all sides (Fig. 2). Circular swimming, for example, could be achieved by suppressing sperm rolling so that the radius of the circular swimming path could result from the intrinsic one-sided asymmetric stroke. Straight-line and curvilinear swimming, perceived as being very distinct motility types and previously associated with, respectively, symmetric and asymmetric controls, are thus potentially closely connected. Both motility types may still be driven by intrinsic asymmetries in their strokes and only differ in how sperm rolling is controlled. The impact of both head spinning and flagellar rolling on the swimming trajectories are yet to be fully explored in the context of sperm steering (*5*).

Tethered sperm experiments are commonly used to study the flagellar beat (*5*, *11*, *50*). Its extrapolation to inform free-swimming behavior has been widely accepted (*5*), driven by the abundance of 2D microscope observations showing straight-line swimming for apparently symmetric side-to-side flagellar movement. However, tethering the sperm suppresses both the head spinning and flagellar rolling that are intrinsic to free-swimming cells. This transforms the 3D asymmetric movement observed here (Fig. 3) into a side-to-side motion for tethered sperm (*5*, *11*, *50*). This substantial discrepancy in flagellar behavior indicates that beating self-organization in sperm is modulated by mechanical constraints imposed on the cell, as has been established for a wide range of flagellar systems (see Supplementary Text). It is therefore difficult to infer free-swimming and rolling behavior from tethered sperm experiments alone (*5*). While 2D observations of tethered sperm have raised questions about the impact of higher beat frequency components on sperm steering (*5*), this does not account for the 3D asymmetric beat in free-swimming and rolling spermatozoa. Future research could investigate whether the higher frequency modes of the 3D beating further regulate the planar and out-of-plane motion–driving sperm rolling to achieve cell steering in 3D. Our 3D observations call into question flagellar control hypotheses (*15*–*18*, *21*) and theoretical/empirical models for sperm swimming and guidance to date (*5*, *6*, *9*, *20*, *43*, *47*, *48*), which ubiquitously assumed either symmetric side-to-side movement in absence of head spinning and sperm rolling, as derived from 2D observations, or idealized helical waveforms with conical symmetry in 3D (see Supplementary Text).

The article "Human sperm uses asymmetric and anisotropic flagellar controls to regulate swimming symmetry and cell steering" was retracted in 2021. Reasons: unreliable data; unreliable results or conclusions.

Computer-assisted semen analysis systems, both in clinics and for research, use 2D views of the sperm’s movement (*2*–*8*, *51*, *52*) and are potentially prone to errors while assessing beating symmetry. 2D projections can introduce low-frequency peaks in the power spectrum of the beat, while averaging out the static mode, due to the sperm rolling motion (Fig. 7F). The spermatozoa of human, bull, and murine species all roll when swimming freely (*4*, *12*, *44*), thus prone to frequency bias in 2D. Planar observations are unable to detect the intrinsic asymmetry of the beat, explaining why this flagellar bias remained invisible until now. Furthermore, symmetry (or the lack of it) is a critical proxy to identify sperm capacitation and hyperactivation, which significantly affect fertility (*10*, *34*, *50*). Despite numerous efforts to capture the flagellar beat in 3D (*12*, *14*, *39*–*41*, *46*, *53*–*58*), the importance of 3D information of the flagellar movement is yet to be fully recognized at the human fertility realm (*51*).

The 3D microscopy and mathematical analysis used here may prove as an essential tool for future studies on the functional nature of both molecular motor asymmetric control and anisotropic signal transduction leading to flagellar self-organization. We hope that these results will motivate further theoretical and empirical investigations on the impact of molecular asymmetries and anisotropies during spontaneous undulations of the flagellar beat in 3D, including comparative investigations among other asymmetric beating–flagellated microorganisms, such as *Chlamydomonas* and murine sperm flagella.

## MATERIALS AND METHODS

### Sperm preparations

Human spermatozoa samples were obtained from healthy donors under written informed consent and with the approval of the Bioethics Committee of the Instituto de Biotecnología, Universidad Nacional Autonoma de México. Human ejaculates were obtained by masturbation after at least 48 hours of sexual abstinence. All human semen samples fulfilled the requirements determined by the World Health Organization. Highly motile sperm were recovered after a swim-up separation for 1 hour in Ham’s F-10 medium at 37°C in a humidified atmosphere of 5% CO_2_ and 95% air. Sperm cells were centrifuged 5 min at 3000 rpm and resuspended in physiological salt solutions at approximately 10^7^ cells/ml. A low viscosity physiological solution was used: 94 mM NaCl, 4 mM KCl, 2 mM CaCl_2_, 1 mM MgCl_2_, 1 mM Na piruvate, 25 mM NaHCO_3_, 5 mM glucose, 30 mM Hepes, and 10 mM lactate at pH 7.4.

The article "Human sperm uses asymmetric and anisotropic flagellar controls to regulate swimming symmetry and cell steering" was retracted in 2021. Reasons: unreliable data; unreliable results or conclusions.

### 3D imaging microscopy

A piezoelectric device P-725 (Physik Instrumente, MA, USA) mounted between a 60× 1.00 numerical aperture water immersion objective (Olympus UIS2 LUMPLFLN 60X W) and an inverted Olympus IX71 microscope, also mounted on an optical table [TMC (GMP SA, Switzerland)], were used. The piezoelectric device oscillates in the vertical direction at 90 Hz with an amplitude of 20 μm and a speed of 3640 μm/s (*53*, *56*, *59*) due to a servo-controller E-501 via a high-current amplifier E-505 (Physik Instrumente, MA, USA). The servo-controller is triggered to vibrate by a ramp signal from the E-506 function generator. A synchronizing transistor-transistor logic pulse from the servo-controller triggers the high-speed camera NAC Q1v with 8-gigabyte random-access memory (recording up to 3.5s at 640 × 480 pixels and 8000 images/s), as further detailed in (*53*, *56*, *59*). Temperature on a Chamlide chamber (CM-B18-1) was controlled at 37°C with a thermal controller (Warner Instruments, TCM/CL-100).

The piezo oscillation, in conjunction with the camera sampling, defines a submicron resolution for the volumetric scan of 0.46 μm. The measured maximum height in the vertical direction between the lowest and highest points of the flagellum for all cells was 14 μm. Thus, the maximum time required to scan the sperm flagellum from the lowest to the highest point is Δ*t_z_* = 3.84 ms. The vertical scan is approximately 65 times faster than the time it takes the sperm flagellum to complete a full revolution around the swimming axis (ω_roll_ = 4 Hz in average for all cells). However, the sperm flagellum continues to move during the volumetric scan, introducing an unavoidable time delay: the time in which the piezo device takes to scan the sperm flagellum in vertical direction Δ*t_z_*. Δ*t_z_* is, however, small when compared with average beating frequency (15 Hz, 66.66 ms per period), equivalent to 5.5% of the beat cycle, while flagella speeds remain below 0.34 μm/ms in 95% of all arc length values recorded in our experimental data. Hence, the maximum flagellar displacement that occurs during the volumetric scan can be estimated by multiplying Δ*t_z_* by all instantaneous flagellar speeds recorded along the arc length. The maximum waveform displacement averaged 0.57 ± 0.37 μm for *s* ≤ 47 μm, where *s* is the flagellar arc length. At the distal region, 47 < *s* < 50 μm, the waveform uncertainty increases to 1.27 ± 0.60 μm. This increase in the distal end is expected from the flagellar tapering of the ultrastructural components toward the submicron scale at this region in mammalian spermatozoa (*2*); thus, this error is intrinsic to any flagellar data capture, including planar waveforms (*2*, *4*, *5*, *47*). As a result, the continuous movement of the flagellum during the volumetric scan introduces distortions in the waveform below the submicron region for *s* ≤ 47 μm and above the one micron region at the distal end for the data reported here. Hence, the time delay introduced by the volumetric scan does not significantly affect the waveform of the flagella. The volumetric scan and the 3D flagellar reconstruction for the spermatozoa in Fig. 2 can be found in movies S1 and S2.

The article "Human sperm uses asymmetric and anisotropic flagellar controls to regulate swimming symmetry and cell steering" was retracted in 2021. Reasons: unreliable data; unreliable results or conclusions.

### Flagella segmentation in 3D

The 3D centerline of the flagellum coordinates was obtained for each 3D stack using a semi-automatic algorithm. For each 3D stack, the flagellum distal point is manually selected from which an automatic algorithm detects the 3D path connecting the sperm head and the selected distal point [Hernandez-Herrera *et al.* (*58*)]. The centroid of the sperm head is used as the initial point to trace the flagellum (3D voxels coordinates), guided by a cost function inversely proportional to the image intensity using a minimal path algorithm, providing the flagellum centerline in 3D voxel coordinates. The 3D spatial coordinates are obtained directly from the microscope pixel resolution and the position of the piezoelectric device. The extracted position of the flagellar coordinates with respect to the laboratory fixed frame of reference, **X**(*s*, *t*) = (*x*, *y*, *z*), is then parametrized by arc length *s* with a total of 100 discretization segments. Data-smoothing routines using the MATLAB “csaps” function were used to remedy random loss of the distal flagellum and remove spatial and temporal noise, as detailed in (*43*). The smoothed data were compared post hoc with the original data to ensure that this process did not cause significant deviations from the original data.

### Human sperm near to and far from the coverslip

We considered a total of 30 human spermatozoa divided into three groups: (a) 20 cells swimming immediately above the coverslip, referred to as sperm “near to” the surface, and with sperm numbers sp1 to sp20; (b) 8 cells swimming with heights between 20 to 85 μm from the surface, referred to as sperm “far from” the coverslip, and with sperm numbers sp21 to sp28; and (c) 2 nonprogressive cells due to the presence of obstacles in their paths immediately above the coverslip and with sperm numbers sp29 and sp30. We define the “free-swimming sperm population” as all spermatozoa that were able to swim freely, groups (a) and (b), totaling 28 cells. The two nonprogressing cells in group (c) are excluded from population averages involving the free-swimming population. The swimming trajectories and flagelloids for each cell are depicted in fig. S4. The heights of each spermatozoa sp21 to sp28 swimming far from the coverslip in group (b) are, respectively, 20, 35, 50, 50, 55, 65, 65, and 85 μm. All spermatozoa investigated here rotated around the rolling axis, including the nonprogressive cells, although the latter rotated in the opposite direction to the free-swimming cells (movies S2 and S6), as detailed in Supplementary Text.

The article "Human sperm uses asymmetric and anisotropic flagellar controls to regulate swimming symmetry and cell steering" was retracted in 2021. Reasons: unreliable data; unreliable results or conclusions.

### Inertia ellipsoids of the flagellum

The total moment of inertia ellipsoid of the flagellum shape is calculated directly from **X**(*s*, *t*), as proposed in (*12*), from which eigenvalues and eigenvectors are calculated to provide the orientation and dimensions of the major, *a*, and minor, *b* and *c*, axis of inertia ellipsoid for each time frame. The ratio *c*/*a* of the inertia ellipsoid captures the three dimensionality of the flagellum in space (fig. S1, B and C) or rather the planarity of the waveform, as if *c*/*a* = 0, then the waveform is a planar curve. The orientation of the major axis of the inertia ellipsoid relative to the solid boundary, located at the plane *z* = 0, defines the angle of attack of the flagellum shape at each instant (fig. S1D).

### The comoving and rolling frame of reference

The 3D flagella coordinate relative to the laboratory fixed frame of reference, **X**(*s*, *t*) = (*x*, *y*, *z*), is transformed into the comoving frame of reference **X***_c_* = (*x_c_*, *y_c_*, *z_c_*) by first translating the waveform relative to the head position and then rotating the waveform around *z* axis so that the mean swimming axis is conveniently aligned with the *x* axis (fig. S3). The comoving frame **X***_c_* is thus the frame of reference translating with the sperm head and rotating with the main swimming axis, as shown in Fig. 2 (B and D) and fig. S3. 3D excursions of the flagella beat induce sperm rolling around the mean axis, defining in this way the “rolling axis” of the flagellum, denoted by the black curve in Fig. 2 (B and D). The comoving frame of reference is transformed into the comoving-rolling frame of reference **X***_cr_* = (*x_cr_*, *y_cr_*, *z_cr_*) by simply rotating the waveform around the rolling axis, taking the angular displacement of mid-flagellar section at the rolling plane as the reference rolling angle (red plane in Fig. 2, B and D, and beating planes illustrated in Fig. 1). That is, no sperm rolling occurs in this reference frame, as shown in Fig. 3E. By construction, the mid-flagellar section of the flagellum is always positioned at the *z_cr_* = 0 with *y_cr_* > 0 at the rolling plane (green plane in Figs. 3E and 4D). Movies S2 to S5 show the flagellar beat for the sperm sp6 in Fig. 3 as seen from the laboratory fixed frame, the comoving frame, and the comoving-rolling frame of references, respectively. The kymographs of the *y* and *z* coordinates in arc length and time for each spermatozoon are shown in figs. S16 to S19 for both frames of reference.

The article "Human sperm uses asymmetric and anisotropic flagellar controls to regulate swimming symmetry and cell steering" was retracted in 2021. Reasons: unreliable data; unreliable results or conclusions.

### PCA of the 3D waveform

We used PCA on the 3D flagellar shape at the comoving, **X***_c_*(*s*, *t*), and comoving-rolling, **X***_cr_*(*s*, *t*), frames of reference. For this, we generalized the previous PCA of scalar quantities (*6*, *18*, *60*) to 3D vectorial functions, in which each spatial coordinate represents an spatiotemporal map in arc length and time (*s*, *t*). With arc length discretized into *m* values, *s*_1_, …, *s_m_*, and time discretized into *n* values, *t*_1_, …, *t_n_*, the augmented matrix for the flagellum coordinates in any generic frame of reference is simply the vector **X***_ia_* = [*x*(*t_i_*, *s*_α_), *y*(*t_i_*, *s*_α_), *z*(*t_i_*, *s*_α_)] and its augmented temporal average is ${\bar{X}}_{i\alpha }=(1/n)\sum_{p=1}^{n}X_{p\alpha }$ for any *i* ∈ {1, …, *n*}. As follows, the eigenvectors of the 3*m* × *m* vectorial covariance matrix, $C_{\alpha \beta }=(1/n)\sum_{i=1}^{n}(X_{i\alpha }-{\bar{X}}_{i\alpha })(X_{i\beta }-{\bar{X}}_{i\beta })$, provide a basis for the 3D flagellar coordinates, with *m* eigenvectors ordered by the size of the associated eigenvalues. Each eigenvector corresponds to a vectorial set of 3D coordinates that define a flagellum shape, also known as PCA modes. Data reconstruction using a simple linear combination of the first two PCA modes is depicted in Fig. 3 (B and F) for, respectively, the comoving and comoving-rolling frames of reference. Mathematically, the PCA reconstruction of the waveform is simply $X_{r}\approx A_{1}(t)X_{\text{pca}}^{1}(s)+A_{2}(t)X_{\text{pca}}^{2}(s)$, where *A*_1_(*t*) and *A*_2_(*t*) are the temporal shape scores for the first $X_{\text{pca}}^{1}(s)$ and second $X_{\text{pca}}^{2}(s)$ PCA spatial modes, respectively. The contribution of each isolated PCA mode on the course of time, $A_{1}(t)X_{\text{pca}}^{1}(s)$ and $A_{2}(t)X_{\text{pca}}^{2}(s)$, defines a surface in space, shown in blue for the first PCA mode and in orange for the second PCA mode in Fig. 3 (C and G), thus depicting the two principal directions of the flagellum beat in 3D for each frame of reference. The PCA reconstruction, PCA modes, and mode amplitudes for each spermatozoon are shown in figs. S6 to S11 for both comoving and comoving-rolling frames of reference.

The article "Human sperm uses asymmetric and anisotropic flagellar controls to regulate swimming symmetry and cell steering" was retracted in 2021. Reasons: unreliable data; unreliable results or conclusions.

### Fourier analysis and traveling wave parameters

We performed Fourier analysis of the spatiotemporal maps of flagellar coordinates at different frames of references, as well as for the curvature and torsion of the waveform. In all cases, the input signal is an undulating wave, generically written as *f* = *f*(*s*, *t*), thus a function of arc length *s* and time *t*. We therefore decompose any generic signal *f* = *f*(*s*, *t*) as a sum of Fourier modes, $f(s,t)=\sum_{n=-\infty }^{\infty }f^{n}(s)\text{exp}\;(\text{in}\omega t)$, where ω is the angular frequency of the signal, ω*_f_*/2π is the signal frequency in cycles per second, *i* is the imaginary number, and *f^n^*(*s*) is the spatial mode indexed by *n*. Each mode *f^n^*(*s*) is a complex-valued function of arc length and captures both the amplitude and the phase of the signal along arc length. The zeroth mode, *n* = 0 of the Fourier spectrum, is referred as the static mode, as its time dependence vanishes, and corresponds to the time average of the signal *f*^0^(*s*) along arc length, denoted in the main text (See the section titled “The human sperm beats anisotropically and asymmetrically”) as superscript 0 of the signal, for example, κ^0^(*s*) is the static mode of the curvature κ. The highest peak in the Fourier spectrum defines the frequency ω*_f_* of the first mode, *n* = 1, also referred as the dynamical mode. The spatiotemporal signal is then approximated by a simple linear combination of the static and dynamic modes, and the signal reconstruction reads *f_r_*(*s*, *t*) ≈ *f*^0^(*s*) + ∣*f*^1^(*s*)∣ sin (ω*t* + ϕ(*s*)), where ∣*f*^1^(*s*)∣ is the amplitude of the dynamical mode and ϕ(*s*) = arg (*f*^1^(*s*)) is the phase of the oscillation, from which the wave parameters may be deduced directly (for example, the rate of decay of the phase along arc length captures the wave speed). Figure 3 (D and H) shows an example of the reconstructed flagellar waveform using the static and dynamic modes of the waveform coordinates, respectively, for the comoving and comoving-rolling frame of references. The black and red curves show, respectively, the individual contributions of the static and dynamic modes (left plot of Fig. 3, D and H), and their sum thus provide the reconstructed waveform (middle plot of Fig. 3, D and H). Low number of periodic cycles may, however, reduce the true intensity of the Fourier transform. This can be mitigated by projecting the Fourier basis on the signal measured directly.

The article "Human sperm uses asymmetric and anisotropic flagellar controls to regulate swimming symmetry and cell steering" was retracted in 2021. Reasons: unreliable data; unreliable results or conclusions.

### Waveform curvature, torsion, and chirality

The tangent, normal, and binormal vectors are calculated directly from flagellum coordinates **X**(*s*, *t*), respectively, via **T** = **X**′, **N** = **T**′/κ and **B** = **T** × **N**, defining the Frenet basis [**T**, **N**, **B**] along arc length *s* at each time *t*, where κ = ‖**T**′‖ and τ = − **N** · **B**′ are, respectively, the 3D curvature and torsion of the flagellum’s centerline. Primes denote derivatives in arc length, *d*/*ds*. Note that the waveform torsion does not capture the mechanical “twist” of the flagellum but rather the 3D turning of the flagellum centerline in space. A purely planar curve embedded in a 3D space has τ = 0. Thus, while the curvature of the waveform captures the actual bending of the flagellum in 3D, the waveform torsion measures the kinematic three dimensionality of the centerline of the flagellum. We also define the “waveform spiral” as the shape of the projection of the waveform in the rolling plane (Fig. 4D), from which the curvature of the spiral, κ*_s_*, can be derived as above. The chirality or handedness (helicity) of the waveform depends on its orientation. For simplicity, the local chiral angle of each section of the flagellum centerline, ψ(*s*_α_, *t*), is defined as the angle between the discrete segment **T**_α_ and the plane defined by **T**_α−2_ × **T**_α−1_ for each flagellar segment *s*_3_, …, *s_m_*, such that if ψ is positive, then the flagellar section is right handed, or if negative, then the flagellar section is left handed (*46*). The magnitude of the discrete angles ψ, however, depends on the number of segments *m*. The kymographs of both *y* and *z* coordinates as a function of arc length and time, and for each spermatozoon, are shown in figs. S16 to S19 for both comoving and comoving-rolling frames of reference. The kymographs of κ, τ, κ*_s_*, and ψ are shown in figs. S20 to S23.

## Supplementary Material

aba5168_SM.pdf

aba5168_Movie_S3.mov

aba5168_Movie_S2.mp4

aba5168_Movie_S1.mp4

aba5168_Movie_S6.mp4

aba5168_Movie_S4.mov

aba5168_Movie_S5.mov

## SUPPLEMENTARY MATERIALS

Supplementary material for this article is available at http://advances.sciencemag.org/cgi/content/full/6/31/eaba5168/DC1

## Appendix

View/request a protocol for this paper from *Bio-protocol*.
